# Study on the Effect of Early Comprehensive Intervention of Skin Contact Combined with Breastfeeding on Improving Blood Glucose in Early Birth of Newborns with Gestational Diabetes Mellitus

This article has been retracted.

**DOI:** 10.1155/2022/2305239

**Published:** 2022-07-31

**Authors:** Xiang Ling, Yan Zhang, Ling Ping Xuan, Jinqi Ma, Wujia Jiang, Yaqin Song, Qian Qian Zhang

**Affiliations:** Wuxi Municipal People's Hospital, Obstetrics 214023, China

## Abstract

**Objective:**

To explore the value of early comprehensive intervention of skin contact combined with breastfeeding on improving early blood glucose in newborns with gestational diabetes mellitus (GDM).

**Methods:**

A total of 300 newborns from pregnant women with gestational diabetes who were hospitalized in Wuxi People's Hospital from January 2021 to December 2021 were randomly assigned into the observation group (*n* = 150) and the control group (*n* = 150). The former group received early comprehensive intervention of skin contact combined with breastfeeding, and the latter group received postnatal naked contact, physical examination after late navel severing, and routine nursing intervention such as early contact and early sucking in 30 min. The peripheral blood microglucose value at 1 and 2 hours after birth, neonatal hospitalization rate, ear temperature of 30 min, 60 min, 90 min, and 120 min after birth, neonatal crying, incidence of postpartum hemorrhage, uterine contraction/wound pain index, lactation before delivery, immediately after delivery, early sucking 15 min, and 2 hours postpartum were observed.

**Results:**

Compared to the control group, the values of trace blood glucose at 1 hour and 2 hours after birth in the observation group were higher, and the difference between groups was statistically significant (*P* < 0.05), the neonatal hospitalization rate in the observation group was lower, and the difference between groups was statistically significant (*P* < 0.05); the ear temperature of 30 min, 60 min, 90 min and 120 min after birth in the observation group was higher, and the difference between groups was statistically significant (*P* < 0.05). The crying frequency of newborns in the observation group was lower, and the difference between groups was statistically significant (*P* < 0.05). The incidence of postpartum hemorrhage in the observation group was lower, and the difference between groups was statistically significant (*P* < 0.05). The rate of uterine contraction/wound pain index grade 1 in the observation group was higher, and the difference between groups was statistically significant (*P* < 0.05). The rates of uterine contraction/wound pain index grade 2 and grade 3 in the observation group were lower, and the difference between groups was statistically significant (*P* < 0.05). The rate of lactation at 2 hours postpartum in the observation group was higher, and the difference between groups was statistically significant (*P* < 0.05).

**Conclusion:**

Early comprehensive intervention of skin contact combined with breastfeeding can significantly increase the early blood glucose of newborns with GDM, effectively promote the occurrence of early hypoglycemia of GDM newborns, avoid a series of serious complications caused by excessive fluctuation of blood sugar, promote the stability of vital signs of newborns, reduce the hospitalization rate of newborns, improve the success rate of breastfeeding, reduce uterine contraction/wound pain, and reduce the incidence of postpartum hemorrhage. My clinical registration number is chictr220059454.

## 1. Introduction

Gestational diabetes mellitus (GDM) not only increases the adverse outcome of pregnancy but also brings many adverse effects on fetal growth and development and neonatal health. The incidence of postnatal hypoglycemia is significantly higher compared to normal newborns [1]. According to the 9th edition of the Global Diabetes Map released by the International Diabetes Federation in 2019, about 16.2% of women around the world give birth to live births with varying degrees of glucose metabolism disorders during pregnancy, of which GDM women account for about 84%. Meanwhile, statistics on the prevalence of GDM in different countries report that the overall prevalence rate of GDM in China is about 8.3% [2]. The incidence of GDM is different in different regions of China. The prevalence rate of GDM in southwest and northwest regions is 4%-5%, while that in densely populated North China, Central China, East China, and South China can be as high as 10% [3]. With the opening of the two-child policy in our country, the rising trend of the prevalence rate of GDM in the whole country is more obvious [4]. As we all know, GDM has adverse effects on the short-term and long-term health of mothers and infants and not only increases the risk of pregnancy infection, polyhydramnios, premature delivery, birth injury, and postpartum infection but also easily leads to neonatal hypoglycemia and other adverse conditions [5].

A report indicates that there is a high incidence of neonatal hypoglycemia in the early postnatal period in pregnant women with GDM, and the incidence of hypoglycemia will increase the risk of neonatal nervous system damage [6–8]. However, there are some problems in clinical hypoglycemia management program of newborn delivered by pregnant women with GDM (infants of diabetic mothers) (hereinafter referred to as IDMS), such as overfeeding, unreasonable blood glucose monitoring, quality standards, and monitoring process which are not standardized. Rationalizing IDMS feeding methods, effective and convenient prevention, and timely treatment of critical hypoglycemia, it is urgent to explore convenient and feasible intervention measures to prevent early hypoglycemia in gestational glucose newborns. Some studies have suggested that skin contact (skin-to-skin contact, referred to as SSC) is beneficial to reduce the incidence of neonatal hypoglycemia, but not enough to improve critical hypoglycemia or hypoglycemia [9]. The strategy guide for promoting breastfeeding points out that healthy newborns and their mothers, early sucking, and early contact newborns have higher levels of 75-180 min blood glucose after birth, but at present, early sucking can be completed in postnatal 30 min-1 h, so it is easy to miss the best dry expectation of IDMS to prevent hypoglycemia, and complicated nursing procedures also increase neonatal bad stress and energy consumption. Some studies have indicated that maternal and infant skin contact with 90 min immediately after birth or longer can simulate the maternal environment for newborns in time, and maternal skin temperature can more effectively reduce the blood sugar consumption caused by newborn's own heat production compared with radiation heating platform [10]. Therefore, this study enrolled 300 newborns from pregnant women with gestational diabetes who were hospitalized in Wuxi People's Hospital from January 2021 to December 2021 and voluntarily participated in this study. Skin contact combined with immediate breastfeeding intervention is expected to enhance the early blood glucose instability of newborns and avoid a series of hazards caused by blood glucose fluctuations and hypoglycemia, which makes blood sugar stable in the ideal state, smooth transition to a relatively safe period, resulting in more social value.

## 2. Patients and Methods

### 2.1. General Information

A total of 300 newborns from pregnant women with gestational diabetes who were hospitalized in Wuxi People's Hospital from January 2021 to December 2021 were randomly assigned into the observation group (*n* = 150) and the control group (*n* = 150). Inclusion criteria are as follows: (1) single and full-term GDM (GDM) newborns; (2) pregnant women over 18-44 years of age; (3) normal uterine development, good health, and singleton; (4) no serious complications and complications during pregnancy, such as severe hypertension, thyroid, liver, and kidney diseases requiring drug treatment; (5) postnatal blood glucose level of 2.2-7.0 mmol/L; (6) effective breastfeeding can be carried out if the amount of breast milk is ≥ (+) within 2 hours after delivery; (7) the information of pregnant women is complete; (8) regular antenatal examination; and (9) informed consent to this study, willing to accept regular follow-up. Exclusion criteria are as follows: (1) pregnant women with cognitive impairment or abnormal behavior; (2) no effective means of contact; (3) prolongation of the first stage of labor and the second stage of labor; (4) cesarean section; (5) excessive fatigue of parturients; (6) no breast milk secretion within 2 hours after delivery; (7) poor nipple condition, newborns cannot suck effectively; (8) moderate and severe neonatal asphyxia; and (9) severe birth injury. Shedding criteria are as follows: (1) those who were asked to drop out of the research or refused to provide relevant information for various reasons or did not give birth in our hospital; (2) participated in other clinical studies during the survey; and (3) during the intervention, the parturient refused to continue to complete the observation index.

### 2.2. Treatment Methods

#### 2.2.1. Technical Route

Technical route is indicated in Figure 1.

#### 2.2.2. Intervention Scheme

The control group was given naked contact after birth, physical examination after late umbilical cord amputation, and routine nursing intervention such as early contact and early sucking within 30 minutes. (1) After GDM pregnant women give birth, medical staff closely observe the delivery process and blood sugar changes of pregnant women in the delivery room, so as to stabilize the pregnant women's emotions and maintain the blood sugar of pregnant women at normal levels; (2) the ambient temperature before delivery is 26-28 degrees, and the preheating temperature of the radiation table is 32-34 degrees. After birth, dry the whole body and head amniotic fluid, lie naked on the parturient's chest, pay attention to the whole body to keep warm, wear a hat, embrace the newborn with both hands, and cover the preheated towel quilt. Meanwhile, umbilical artery blood was taken for blood glucose monitoring for the first time. Newborns with postnatal blood glucose level of 2.2-7.0 mmol/L were enrolled in the observation group; (3) newborns after late umbilical cord amputation were routinely treated with umbilical cord and physical examination in the rewarming table and wrapped to keep warm after no abnormalities. Mother-to-infant skin contact and crawling breast search were carried out in 30-60 min; (4) if the postnatal umbilical artery blood glucose was higher than 2.6 mmol/L, the heel blood samples were collected at 1 hour and 2 hours after delivery to detect the peripheral blood glucose value after routine intervention; (5) those with blood sugar 2.2-2.6 mmol/L immediately after birth should be regularly fed with 10% glucose solution 10 mL/kg or infant formula 10 mL/kg when opening milk. The peripheral blood glucose was measured again at 30 and 60 minutes after intervention, and the blood glucose after intervention was lower compared to that after 2.2 mmol/L transfer to pediatrics.

The scheme of the observation group is as follows: the observation group received early comprehensive intervention of skin contact combined with breastfeeding. (1) Routine nursing: on the basis of the treatment in the control group, the mothers and newborns were exposed to at least 90 min immediately after birth, and the biological nursing method was employed to assist the pregnant women and newborns to breastfeed immediately during the complete skin contact between the mothers and newborns. Among them, in biological breastfeeding strategy, when the mother is breastfeeding, both the mother and the newborn are in a relaxed posture, the lying or semisitting position; the head, neck, shoulder, and waist can be well supported. The newborn lies prone on the mother's chest, and the two bodies can fit closely under the action of gravity, from the whole area of the body from the sternum to the pubic bone, and the thigh of the newborn. Calves and tiptoes are spontaneously applied to the maternal body or part of the environment (beds, sofas, chairs, clothes on the bed, etc.), and newborns can fix themselves without too much help. There is no need for the woman to exert too much pressure on the head and back, which is easier to breathe and does not need to change positions too much. This method is helpful to stimulate the natural lactation and foraging behavior of parturients and newborns. Newborns approach the breast and take the initiative to make the head swing vertically and the limbs and body swing together and finally achieve independent milk. (2) Treatment of neonatal hypoglycemia: on the basis of treatment in the control group, complete skin contact between mother and infant combined with breastfeeding continued after each formula feeding. (3) Treatment of neonatal critical hypoglycemia: continuous complete skin contact between mother and infant and breast feeding in biological position. The peripheral blood glucose was measured again at 30 and 60 minutes after intervention, and the blood glucose after intervention was lower than that after 2.2 mmol/L transfer to pediatrics.

### 2.3. Observation Index

The main results were as follows:

1. The values of trace blood glucose in peripheral blood at birth and 1 hour and 2 hours after birth were observed. The normal value of blood glucose within 24 hours after birth was 2.2-7.0 mmol/2.6 mmol/L, and the critical blood glucose value was 2.2 mmol
2. To observe the hospitalization rate of neonatal pediatrics. Neonatal pediatrics hospitalization rate = the number of newborns transferred to neonatal pediatrics due to hypoglycemia/the total number of newborns in the group × 100%
3. To observe the ear temperature of 30 min, 60 min, 90 min, and 120 min after birth, the ear temperature of 30 min, 60 min, 90 min, and 120 min was measured and recorded by the midwife immediately after birth and immediately after birth. The normal ear temperature of the newborn was 36.5~37.5°C
4. The crying of newborns in the two groups was observed. Record one continuous crying, and record the next one if the crying interval is 3 minutes or more
5. The incidence of postpartum hemorrhage and uterine contraction/wound pain index was observed. Refer to the pain grade prescribed by the World Health Organization (WHO): grade 0 (painless): no pain, can be accompanied by mild discomfort; grade 1 (mild): slight pain; grade 2 (moderate): obvious pain, with sweating and dyspnea; and grade 3 (severe): severe pain, unbearable
6. The milk yield of the two groups was observed before delivery, immediately after delivery, 15 minutes after early sucking, and 2 hours after delivery. Evaluation criteria of breast milk volume are as follows: 1 min artificial milking method was adopted to evaluate the amount of milk with naked eyes, no milk was extruded as (-), 1 drop or 2 drops was extruded as (+), milk could flow out continuously as (+ +), milk could flow out more or ejected out as (+), (-) and (+) represented insufficient breast milk, and (+) and (+) represented sufficient breast milk

### 2.4. Statistical Analysis

The statistical analysis of the data in this study uses SPSS24.0 software, and the statistical graphics are drawn by GraphPad Prism 8.0. The measurement data in accordance with normal distribution were presented by mean ± standard deviation, paired sample *t*-test was employed for intragroup comparison, and independent sample *t*-test was adopted for intergroup comparison. If not, it is expressed by median (lower quartile to upper quartile), paired sample nonparametric test is employed for intragroup comparison, and independent sample nonparametric test is adopted for intergroup comparison. The grade data were tested by FISHER accurate method. *P* < 0.05 indicated that there exhibited statistical significance.

## 3. Results

### 3.1. To Observe the Value of Trace Blood Glucose in Peripheral Blood of Newborns in Both Groups at 1 h and 2 h after Birth

The values of trace blood glucose at 1 hour and 2 hours after birth in the observation group were higher compared to the control group, and the difference between groups was statistically significant (*P* < 0.05). As indicated in Table 1.

### 3.2. To Observe the Hospitalization Rate of Neonatal Pediatrics in Two Groups

The neonatal hospitalization rate in the observation group was lower compared to the control group (*P* < 0.05), as indicated in Table 2.

### 3.3. To Observe the Ear Temperature of 30 min, 60 min, 90 min, and 120 min after Birth in Two Groups of Newborns

The ear temperature of 30 min, 60 min, 90 min, and 120 min of newborns in the observation group was higher compared to the control group, and the difference between groups was statistically significant (*P* < 0.05), as indicated in Table 3.

### 3.4. To Observe the Crying of Newborns in Two Groups

The crying frequency of newborns in the observation group was lower compared to the control group, and the difference between groups was statistically significant (*P* < 0.05), as indicated in Table 4.

### 3.5. The Incidence of Postpartum Hemorrhage and Uterine Contraction/Wound Pain Index Were Observed between the Two Groups

The incidence of postpartum hemorrhage in the observation group was lower compared to the control group, and the difference between groups was statistically significant (*P* < 0.05). The rate of uterine contraction/wound pain index grade 1 in the observation group was higher compared to the control group, and the difference between groups was statistically significant (*P* < 0.05). The rates of uterine contraction/wound pain index grade 2 and grade 3 in the observation group were lower compared to the control group, and the difference between groups was statistically significant (*P* < 0.05), as indicated in Tables 5 and 6.

### 3.6. To Observe the Lactation of the Two Groups 2 Hours after Delivery

The rate of lactation (+++) at 2 hours postpartum in the observation group was higher compared to the control group, and the difference between groups was statistically significant (*P* < 0.05), as indicated in Table 7.

## 4. Discussion

Gestational diabetes mellitus (GDM) refers to different degrees of abnormal glucose metabolism in women during pregnancy or found for the first time [11]. The maternal blood glucose level of pregnant women with GDM is high, which causes a large amount of glucose to enter the fetus through the placenta, and the fetal blood glucose level also increases [12]. The increase of blood glucose level can stimulate the compensatory proliferation of fetal islet cells and produce more insulin than needed [13]. After the delivery of newborns, the storage of glycogen in the body is insufficient, and the newborns delivered by pregnant women with GDM tend to have heavy body weight, resulting in an increase in glucose metabolism and consumption and a significant increase in the incidence of neonatal hypoglycemia after birth [14]. Hypoglycemia can make the energy source of neonatal brain cell metabolism insufficient, and brain metabolism and other physiological activities cannot be carried out normally [15]. If neonatal hypoglycemia cannot be treated in time, it may cause irreversible brain damage [16, 17].

Maintaining the dynamic stability of blood glucose is an important physiological link in the transition from fetus to newborn. Studies have indicated that the lower the blood sugar and the longer the duration, the greater the likelihood of brain injury [18]. Regardless of gestational age and age, whole blood glucose < 2.2 mmol/L was diagnosed as neonatal hypoglycemia, and when blood glucose < 2.6 mmol/L, it was critical hypoglycemia, and clinical intervention was needed. Whether brain injury occurs in children with hypoglycemia is not only related to the previously recognized lowest blood glucose level and duration of hypoglycemia but also related to blood glucose variation indexes such as maximum blood glucose fluctuation, standard deviation of blood glucose level, and average blood glucose fluctuation [19]. It is suggested that the blood glucose level should be closely monitored in the process of clinical treatment of hypoglycemia, and the speed of correcting hypoglycemia should not be too fast and the range should not be too high. Early intervention in clinical work is expected to reduce a series of hazards caused by hypoglycemia [20].

In 2019, a study on the integration of clinical nursing practice guidelines for GDM pointed out that the blood glucose level of newborns should continue to be higher than 2.5 mmol/L within 24 hours after birth. Studies have indicated that the most obvious decrease in blood glucose in newborns with IDMS is within 0.5 hours after birth, and it is also an important period to prevent hypoglycemia [21]. Blood glucose in 2-48 hours after birth of IDMS indicates an upward trend. Transient hypoglycemia is common during this period, and because newborns can tolerate hypoglycemia to a certain extent, there may be a lack of typical clinical symptoms in the early stage [22]. According to the American Academy of Pediatrics, blood glucose monitoring should be performed routinely in children with high-risk factors for hypoglycemia. A study found that the study monitored the blood sugar of newborns who were not fed for 3 hours and found that the blood sugar was the lowest within 1-2 hours and increased after 3 hours [23]. Studies have indicated that there is a tendency to maintain blood glucose in the normal range with the continuous improvement of the mechanism of blood glucose regulation by IDMS and reasonable feeding.

At present, China has not formulated guidelines for the management of neonatal hypoglycemia, and the diagnosis of neonatal hypoglycemia basically follows the previous clinical or epidemiological definition [24]. When newborns develop critical hypoglycemia, they are often fed with 10% glucose or formula. The clinical management model of neonatal hypoglycemia has a standardized management mode, which is limited to monitoring blood glucose value on the basis of early breastfeeding, while 10%GS or formula intervention is the main line [25]. The improved scheme cannot reduce the incidence of postnatal 30 min hypoglycemia, which has some limitations. Studies have indicated that the osmotic concentration of 10% GS > 400 mmol/L will damage the intestinal mucosa of newborns and lead to necrotizing enterocolitis; although the osmotic concentration of formula is less than 400 mol/L, the rapid increment will also lead to intestinal mucosal damage of newborns [26].

Breast milk is considered to be the most ideal food to prevent neonatal hypoglycemia. Continuous breastfeeding and frequent sucking of newborns can promote their sympathetic adrenaline stress response, which in turn leads to an increase in blood sugar. The Breastfeeding Promotion Strategy Guide points out that healthy newborns and their mothers and babies with early sucking and early contact have higher 75-180 min blood glucose levels after birth [27]. SSC nursing is a new nursing mode and it is when a newborn is born or shortly after birth, causing it to touch naked on the mother's naked chest. The peripheral receptors of newborns are stimulated by skin contact, and the signals are transmitted by neurons to the tactile, motor sensory system, and vestibule, respond when the signal is received, effectively adjust the movement state of the human body, and relieve stress response [28]. Rongjin et al. have studied the SSC proposed which is helpful to reduce the incidence of neonatal hypoglycemia [29]. At present, the first clinical breastfeeding is completed within 30-60 min after birth, or crawling is used to complete the first early sucking, but it is not clear whether early breastfeeding of IDMS can be completed in advance. Therefore, this paper carried out a study to explore the value of early comprehensive intervention of skin contact combined with breastfeeding on improving early blood glucose in neonates with GDM.

The results of this study indicated that after the early comprehensive intervention of skin contact combined with breastfeeding, the peripheral blood glucose at 1 hour and 2 hours after birth, and the ear temperature of 30 min, 60 min, 90 min, and 120 min after birth, lactation rate (+++) at 2 hours postpartum was higher compared to routine intervention (*P* < 0.05). Neonatal hospitalization rate, neonatal crying frequency, incidence of postpartum hemorrhage, uterine contraction/wound pain index grade 2 and grade 3 were lower than those of routine intervention (*P* < 0.05) [30]. It is proved that the early comprehensive intervention of skin contact combined with breastfeeding is helpful to stabilize the early blood glucose and body temperature of newborns, promote breast milk secretion, avoid neonatal crying and uneasiness, reduce the hospitalization rate of neonatal hypoglycemia, and reduce the incidence of postpartum hemorrhage. This is mainly because a number of research reports pointed out that hypothermia is an important risk factor for neonatal hypoglycemia [30, 31]. Due to the great changes in environmental temperature after birth, newborns need a large amount of sugar energy to be converted into calories to maintain body temperature, and energy consumption has increased significantly. However, traditional breastfeeding and skin contact are usually performed after the completion of routine neonatal nursing operations, such as umbilical cord ligation and measurement of body mass and body length. At this stage, the maternal glucose supply is interrupted, the stimulation of the new environment triggers anaerobic metabolism and consumes a lot of blood sugar, and the energy consumption is also increased by the change of ambient temperature and crying after delivery [31]. On the one hand, timely and good temperature transfer can effectively increase newborn body temperature, avoid neonatal crying, reduce extra energy consumption, and avoid hypoglycemia [32–34]. Meanwhile, it can increase the time of neonatal breastfeeding and the success rate of breastfeeding and increase the amount of maternal lactation [35]. The studies of Feng et al. indicated that newborns were in a quiet awakening or sleeping state most of the time during mother-to-infant skin contact, and the number of crying and the duration of crying decreased significantly. It plays an effective positive role in regulating the behavior of newborns [36]. The qualitative research of Yufeng indicates that the pregnant woman is full of satisfaction and pleasure when the mother is in complete skin contact, which is a kind of physical and mental pleasant experience, and establishes the mother's sense of responsibility as soon as possible and promotes maternal spontaneous breastfeeding and soothing newborn behavior [37]. On the other hand, biological rearing, also known as semilying lactation, was first recorded by Klaus and Kennel (1976) [38, 39]. Babies release innate reflexes and mothers release instinctive behavior. Both mothers and newborns can be in a relatively relaxed position during breastfeeding. The newborn lies prone on the mother's bare chest, and the body is close to the mother and can be supported and fixed from the mother's body and surrounding environment. The mother can hold the newborn frequently for a long time, find the feeding reaction of the newborn in time, breastfeed in time, and provide energy, which can well solve the problems of energy consumption, crying, and not keeping warm in time [40]. And it can enhance the effective sucking rate of newborns, promote uterine contraction, reduce the amount of postpartum bleeding as well as the feeling of uterine contraction/wound pain, and strengthen the overall intervention effect. There are some limitations in this study. First, the sample size of this study is not large and it is a single-center study, so bias is inevitable. In future research, we will carry out multicenter, large-sample prospective studies, or more valuable conclusions can be drawn.

Conclusively, early comprehensive intervention of skin contact combined with breastfeeding can significantly increase the early blood glucose of newborns with GDM, effectively promote the occurrence of early hypoglycemia of GDM newborns, avoid a series of serious complications caused by excessive fluctuation of blood sugar, promote the stability of vital signs of newborns, reduce the hospitalization rate of newborns, improve the success rate of breastfeeding, reduce uterine contraction/wound pain, and reduce the incidence of postpartum hemorrhage.

## Figures and Tables

**Figure 1:** Technical route.

**Table 1:** Comparison of peripheral blood glucose values in two groups of newborns at 1 hour after birth.

Grouping	The value of trace blood glucose in peripheral blood at 1 hour after birth (mmol/L)	Trace blood glucose value of peripheral blood 2 hours after birth (mmol/L)
Control group (*n* = 150)	3.44 ± 0.11	3.34 ± 1.11
Observation group (*n* = 150)	3.71 ± 0.26	3.74 ± 1.18
*t* value	11.713	3.024
*P* value	<0.05	<0.05

**Table 2:** Comparison of the hospitalization rate of neonatal pediatrics in two groups.

Grouping	The number of newborns transferred to neonatal pediatrics due to hypoglycemia (example)	Neonatal pediatrics hospitalization rate (%)
Control group (*n* = 150)	15	10.00
Observation group (*n* = 150)	5	3.33
*χ* ^2^ value	5.357	
*P* value	<0.05	

**Table 3:** Comparison of the ear temperature of 30 min, 60 min, 90 min, and 120 min after birth in two groups of newborns.

Grouping	Ear temperature of 30 min after birth (°C)	Ear temperature of 60 min after birth (°C)	90 min ear temperature after birth (°C)	Ear temperature of 120 min after birth (°C)
Control group (*n* = 150)	36.54 ± 0.09	36.32 ± 0.03	36.33 ± 0.12	36.41 ± 0.21^∗^
Observation group (*n* = 150)	36.85 ± 0.02	36.72 ± 0.17	36.75 ± 0.08	36.85 ± 0.06^∗^
*t* value	41.181	28.038	35.667	24.674
*P* value	<0.05	<0.05	<0.05	<0.05

**Table 4:** Comparison of the crying of newborns in two groups.

Grouping	Neonatal crying (times/h)
Control group (*n* = 150)	8.15 ± 1.45
Observation group (*n* = 150)	5.16 ± 0.88
*t* value	21.590
*P* value	<0.05

**Table 5:** Comparison of the incidence of postpartum hemorrhage in two groups.

Grouping	Postpartum hemorrhage (example)	Incidence of postpartum hemorrhage (%)
Control group (*n* = 150)	13	8.67
Observation group (*n* = 150)	2	1.33
*χ* ^2^ value	8.491	
*P* value	<0.05	

**Table 6:** Comparison of uterine contraction/wound pain index between the two groups.

Grouping	Level 0 (example (%))	Level 1 (example (%))	Level 2 (example (%))	Level 3 (example (%))
Control group (*n* = 150)	0/0.00	42/28.00	51/34.00	57/38.00
Observation group (*n* = 150)	0/0.00	74/49.33	35/23.33	41/27.34
*χ* ^2^ value		14.393	4.173	3.879
*P* value		<0.05	<0.05	<0.05

**Table 7:** Comparison of lactation 2 hours after delivery in two groups.

Group	Milk yield at 2 hours postpartum +++ (example)	Milk yield at 2 hours +++ proportion (%)
Control group (*n* = 150)	120	80.00
Observation group (*n* = 150)	142	94.67
*χ* ^2^ value	14.584	
*P* value	<0.05	

## Data Availability

No data were used to support this study.
